# Enhancing data security and privacy in energy applications: Integrating IoT and blockchain technologies

This article has been retracted.

**DOI:** 10.1016/j.heliyon.2024.e38917

**Published:** 2024-10-05

**Authors:** Hari Mohan Rai, Kaustubh Kumar Shukla, Lilia Tightiz, Sanjeevikumar Padmanaban

**Affiliations:** a School of Computing, Gachon University, 1342 Seongnam-daero, Sujeong-gu, Seongnam-si, 13120, Gyeonggi-do, Republic of Korea; b Department of ECE, Dronacharya Group of Institutions, Greater Noida, India; c Department of Electrical Engineering, IT and Cybernetics, University of South-Eastern Norway, Porsgrunn, 3918, Norway

**Keywords:** Blockchain, Internet of things (IoT), Nuclear energy, Data security, Data privacy, Cryptographic transactions, Secure data management framework, IoT-blockchain integration

## Abstract

The integration of blockchain technology with the IoToffers numerous opportunities to enhance the privacy, security, and integrity. This study comprehensively analyze the challenges, scope, and potential solutions associated with integrating blockchain technology and the IoT, with a specific emphasis on nuclear energy applications. We discuss the roles and various aspects of blockchain and the IoT, highlighting their multiple dimensions and applications. Our study develops a secure data management framework that incorporates encryption, integrity verification, an integrated communication network, and a robust data flow architecture. We explore the several aspects of data security, privacy, and integrity, along with the potential solutions in the integration of blockchain and IoT. The study also investigates the secure transaction process, with a specific focus on cryptographic, mathematical, and algorithmic perspectives. We demonstrated the use of blockchain technology in the nuclear energy sector using flow charts, comprehensively addressing the associated security and privacy concerns. While emphasizing the applicability of our methodology to the nuclear sector, we also acknowledge limitations such as requirements for practical validation, challenges with resource-constrained IoT environments, increasing cyberthreats, and limited real-time data availability. The future scope of our study focuses on standardization, scalable blockchain, post-quantum cryptography, privacy, regulations, real-world testbeds, and deep learning for nuclear sector security. Our findings highlight that the integration of blockchain and IoT can significantly enhance the security and privacy of nuclear energy applications, although practical validation and optimization are necessary.

## 1 Introduction

The digital age has made security and privacy imperative, particularly with the growth of IoT and blockchain technology [1]. Security keeps confidence high, guarantees system integrity, and guards sensitive data including financial and personal information. People who value privacy are able to freely express themselves, take control of their digital footprint, and are shielded from discrimination. Security and privacy issues are brought up by the IoT's massive network of linked devices. Even with its robust security features, blockchain still has privacy issues to deal with [2].

A safer and more reliable online environment may result from awareness of and adherence to these fundamental rights. With features like immutability, decentralization, and transparency, blockchain technology is a shared ledger that logs transactions via a network of computers [3]. In IoT settings, sensor data from devices may be safely kept on a blockchain, where each block is cryptographically connected to the one before it. As a result, the integrity and dependability of the data gathered are guaranteed and a tamper-proof record of transactions is produced. Additional benefits of blockchain include improved access control, which guards user privacy and stops illegal data breaches. By doing away with the requirement for a central authority, it also promotes decentralized trust and lowers the risk of security breaches.

Although there are still issues with scalability and privacy, blockchain technology is a viable solution for protecting and handling data on the IoT [4].

The IoT is a network of interconnected objects that gather and share data via the internet, such as industrial machines, refrigerators, and thermostats [5]. Known as "smart objects," these gadgets have the ability to automate processes, increase energy efficiency, and offer security features. Applications for IoT are numerous and constantly growing; Industrial IoT (IIoT) is centered on lowering costs and increasing efficiency [6,7]. However, because gadgets are networked, security and privacy issues become relevant. IoT has enormous promise in the future and it will only get bigger [8].

Fig. 1 shows the IoT block diagram, which comprises of an Arduino or Raspberry Pi, an IoT board, and a sensor module. Program dumps utilizing the Serial Communication Protocol or I2C may be made using the Arduino Suite [9]. Radio waves are sent by an RF module. Web-based user interfaces and Virtual Private Servers (VPS) must be used for network setup. IoT servers collect and monitor data, which is then safely stored in big data analytics [10,11].

**Fig. 1:** IoT system with sensor data acquisition and cloud storage.

Blockchain technology and the IoT offer a promising future for secure and private data management. Blockchain's immutability, transparency, and decentralization address security and privacy concerns in IoT systems [9]. It provides tamper-proof data, fosters decentralized trust, and allows for granular access control. However, challenges include scalability and privacy-preserving techniques [12]. Traditional blockchain implementations are resource-intensive, and lightweight protocols are being explored for low-power devices. As research progresses, more robust and scalable solutions will unlock the full potential of blockchain in IoT data management [13]. Blockchain technology, first introduced in 2008 to address double spending in digital cash, has since gained popularity for its security, immutability, traceability, and transparency [14]. Initially used to support BITCOIN transactions, blockchain has become widely adopted by governments, businesses, and organizations due to its efficient and secure nature. It is composed of blocks linked together, providing a highly distributed ledger for transaction keeping, auditing, and recording [15]. The genesis block is the first hashed block on the blockchain, recording the first transactions. It is linked to every subsequent block by a unique hash. Blockchain confirms transaction validity through consensus, validating transactions across nodes [16]. It offers transparency, traceability, and security, making it a secure, non-mutable linear chaining system. Blockchain simplifies transaction storage and asset tracking in business networks [17].

While a basic blockchain workflow involves collecting transactions, grouping them into blocks, hashing those blocks, verifying them, and adding them to the chain [18], Fig. 2 delves deeper into this process for a generic blockchain system. The journey starts with users initiating transactions on the network [19]. These transactions are then collected and temporarily stored in a pool. Miners or validators, depending on the system, select transactions from this pool and meticulously validate them (e.g., verifying signatures). Once validated, these transactions are included in a newly created block. This newly minted block doesn't get added to the chain straightaway. It's broadcasted across the network, where individual nodes independently verify the block's legitimacy. This verification process involves several steps: ensuring the validity of individual transactions (e.g., verifying signatures), confirming the hash of the previous block in the chain, and guaranteeing adherence to the consensus mechanism rules (e.g., proof-of-work). If a sufficient number of nodes agree on the block's validity through the consensus mechanism, it's considered confirmed. These confirmed blocks are then permanently etched into the distributed ledger, a replicated database maintained by all participants on the network [20]. It's important to note that some blockchain systems utilize transaction fees to incentivize miners or validators. These fees might be handled in a separate step, where transactions with insufficient fees are rejected and returned to the pool for another attempt. The type of permissioned access to the blockchain network can influence the level of trust and classification associated with it [21]. There are some common blockchain network types, Open networks where anyone can participate in the consensus process, offering complete transparency but potentially facing scalability challenges due to the sheer number of participants [21]. Closed networks with restricted access controlled by a central authority, providing increased scalability and transaction speed at the cost of reduced decentralization and trust. Permissioned networks where a pre-selected group of organizations participate in the consensus process, striking a balance between security, scalability, and control. These combine elements of public and private blockchains, offering flexibility in access control and functionalities. By understanding the detailed transaction flow and the different network types, we gain a deeper appreciation for the intricacies and versatility of blockchain technology.

**Fig. 2:** Detailed workflow of a generic blockchain system.

Blockchain technology offers numerous benefits for security and privacy use cases [22]. It provides resilience and availability, reducing the risk of threats, corruption, and disruption. Decentralized infrastructure reduces data exposure and redundancy, making security decisions closer to the network's periphery [23]. Blockchain data is tramper proof, ensuring transactions are validated by consensus. Distributed ledger and blockchain designs are emerging as viable solutions for distributed governance, healthcare, data provenance, and cross-institutional collaboration [24]. Blockchain technology also offers transparency and traceability, storing entire transaction data as tamper-proof records, reducing the possibility of counterfeiting and tampering [25]. It can make remittances and cross-border payments safer and more private. Blockchain can also be used for identity and authorization, preventing attacks in the supply chain life cycle, especially for edge IoT devices. Blockchain technology also provides identity protection, authentication, access management, and proof of ownership [26]. It makes it difficult to alter information stored on-chain, guarantees privacy, and prevents single-point failure proof through decentralized multi-signature base administration systems [27]. In early 2000, Kevin Ashton introduced the concept of the IoT to Procter and Gamble. IoT devices, including wireless sensors, actuators, and computers, exchange data through the internet [28]. These web-enabled embedded systems process, sense, and communicate data from their environments, connecting to gateways for analysis. IoT devices are designed to perform work without human intervention and depend heavily on IoT applications [17].

The IoT enables people to live and work smartly, making businesses and industries smarter and more manageable. It also automates processes, reduces manual labor costs, and improves facility distribution. IoT devices, classified based on communication type, enable public or multitenant networks to connect multiple applications [29]. They are capable of small payloads, long intervals, battery power, and low latency. IoT standards include IPv6, Bluetooth Low Energy (BLE), Z-Wave, 804.15.4, 6LoWPAN, ZigBee, LiteOS, OneM2M, Data Distribution Service (DDS), Advanced Message Queuing Protocol (AMQP), Constrained Application Protocol (CoAP), and Long Range Wide Area Network (LoRaWAN). IoT connects billions of devices to the internet and streams data, but security and privacy are major concerns due to increased attack surface [30]. IoT devices can be exploited by hackers to exploit weaknesses in devices and make them unusable. Privacy is a major concern for IoT users, and IoT threatens critical infrastructures like electricity, transportation, and financial services [31]. An IoT ecosystem consists of internet-enabled devices that use systems on a chip to collaborate. Processors and sensors act as transmitters and receivers, transmitting and gathering data from their environments [32]. IoT applications' connectivity, networking, and communication protocols depend heavily on collaboration, and artificial intelligence and machine learning can improve data-gathering processes [33,34]. IoTs enable businesses, industries, and personal life to become smarter by providing connected devices, automating processes, and providing real-time analytics [35]. Building on recent advances in decision-making methodologies and data integration techniques, as presented by Mondal & Roy (2024) [36] in their work on Fermatean fuzzy Mahalanobis distance for supply chain management and Debnath & Roy (2023) [37] in the application of T-spherical fuzzy sets in refueling site selection, this study aims to address significant challenges in secure data management through the integration of IoT and Blockchain technology.

Strong security measures are urgently required as demonstrated by our increasing dependence on networked systems and the volume of sensitive data that is growing. Although blockchain technology presents significant challenges when integrating with Internet of Things devices, it provides new opportunities to enhance data integrity and transparency. This study is motivated by the need to bridge this gap and create a thorough framework for safe data handling in industries that depend on vital infrastructure, including nuclear energy. The aim of this study intends to develop secure and resilient systems by addressing the limitations of present approaches and exploring the potential benefits for the integration of the blockchain and IoT.

## 2 Literature review

The integration of blockchain technology with the IoT has garnered significant attention in recent years, with researchers exploring various approaches to address challenges and exploit advantages in different domains. The reason of this integration is to address the many challenges such as data privacy, security, integrity and scalability, these are the vital in IoT environments described by substantial networks of interconnected devices. The varios studies by many researchers explored the applications of blockchain in many domains such as healthcare, supply chain, industry, smart city, telecommunications, e-Voting, etc, with focuses on increasing the security issues and the reliability of IoT systems. In supply chain management [22,[38], [39], [40]], blockchain is being controlled to ensure integrity and traceability, enabling real-time monitoring of goods as they passage through complex global network. Blockchain in healthcare [[41], [42], [43], [44]], utilized to secure the patient data, insuring the privacy and integrity of the patents data, also secure data sharing across organizations. Additionally, smart cities [16,45] are also implementing blockchain to govern and improve metropolitan infrastructure, from energy grids to public transportation systems, by ensuring data integrity and enabling decentralized decision-making.

Table 1 encompasses diverse approaches and their focuses on integrating IoT and Blockchain across various applications, along with the findings and limitations. During our review, we utilized several peer-reviewed literatures published during 2017–2024. Based on the insights gathered from the table, we present our observations.

**Table 1:** A Review of IoT and blockchain integration across domains.

Reference	Authors	Year	Focus	Advantages	Limitations
[5]	A. Dorri	2017	Optimization of blockchain for IoT	Optimizing blockchain technology for efficient and cost-effective use in IoT applications.	Trade-off between scalability and security, potential for vulnerabilities in the underlying consensus mechanisms.
[1]	(Sagirlar et al.	2018	Hybrid blockchain architecture for IoT	Scalable and decentralized infrastructure for secure data exchange in IoT networks.	Increased complexity compared to traditional architectures, potential for scalability bottlenecks at high transaction volumes.
[14]	A. F. Zorzo et al.	2018	Dependable IoT using blockchain	Utilizing blockchain to ensure data integrity and fault tolerance in IoT systems.	Scalability challenges and potential for network congestion as the number of devices increases.
[38]	S. Aich et al.	2019	Benefits of blockchain in supply chain	Enhancing transparency, traceability, and reducing fraud in supply chain management with blockchain.	Integration challenges between existing systems and potential privacy concerns regarding data visibility.
[22]	A. Rejeb et al.	2019	Leveraging IoT and blockchain in SCM	Combining IoT and blockchain to improve supply chain visibility and reduce costs	Increased complexity in implementation and potential interoperability issues between different systems.
[46]	T. Alam	2019	Role of blockchain in IoT	Leveraging blockchain for data integrity, transparency, and decentralized control in IoT systems.	Potential scalability limitations and increased energy consumption compared to centralized approaches.
[45]	L. T. Khrais	2020	Role of IoT and blockchain in smart city	Utilizing IoT and blockchain to enhance data security and improve efficiency in smart city applications	Integration challenges between various systems and potential privacy concerns regarding collected data.
[47]	D. Pavithran	2020	Blockchain framework for IoT	Developing a blockchain framework for secure and reliable data management in IoT networks.	Scalability limitations and potential performance bottlenecks as the network grows.
[41]	P. Hemalatha et al.	2021	Monitoring and securing healthcare data	Enabling tamper-proof healthcare data records and enhanced security through blockchain technology.	Privacy concerns regarding sensitive health data and potential regulatory hurdles in healthcare data management.
[48]	E. A. Shammar and A. T. Zahary	2021	Security perspective of IoT integration	Enhancing data security and reducing fraud risk through blockchain integration with IoT systems.	Increased complexity and potential performance overhead due to the distributed nature of blockchain.
[43]	Kumaresan et al., 2022	2022	Blockchain, IoT, and 5G in smart healthcare	Leveraging the combined benefits of blockchain, IoT, and 5G technology to improve security and privacy in smart healthcare systems.	Integration challenges between these disparate technologies and potential scalability issues.
[49]	Alzuabi et al.	2022	Privacy and security issues in blockchain-based IoT systems	Identifying and addressing privacy and security vulnerabilities in blockchain-based IoT systems.	Balancing privacy concerns with the need for data transparency and potential security exploits in the underlying blockchain technology.
[50]	Santos et al.	2023	Blockchain-based loyalty management	Utilizing blockchain to incentivize customer loyalty and reduce costs in loyalty programs.	Requirement for a generic platform to facilitate widespread adoption and potential integration challenges with existing systems.
[51]	Sallal et al.	2023	Privacy and verifiability in e-voting	Achieving both privacy and verifiability in electronic voting systems using cryptographic primitives enabled by blockchain.	Increased complexity due to cryptographic techniques and potential usability challenges for voters.
[52]	Magara & Zhou	2024	Examination of IoT applications and privacy/security concerns	Analyzing privacy and security risks associated with various IoT applications and proposing scalable.	Difficulty in implementing effective solutions and adapting existing policy frameworks to address the evolving nature of IoT threats.
[42]	T. Wang et al.	2024	Revolutionizing Healthcare Data Sharing using Secure Hybrid Blockchain Approach	Unlocking the Power of Secure and Private Health Data Exchange.	Navigating the Intricacies: Implementation Complexity and Potential Scalability Hurdles.

Dorri (2017) [5] tackles the crucial issue of optimizing blockchain for resource-constrained IoT environments. This approach aims to overcome limitations in scalability and efficiency by tailoring the blockchain architecture specifically for IoT use cases. Sagirlar et al. (2018) [1] promoted a hybrid strategy that makes use of the advantages of both private and public blockchains. For IoT applications, this approach promotes security, decentralization, and scalability. On the other hand, handling the complexities of Proof-of-Work sub-blockchains requires careful consideration. Zorzo et al. (2018) [14] explored the blockchain's possibility of building trustworthy IoTsolutions. Their primary focus is on data integrity and reliability, which are essential components for critical systems that depend on information that is reliable. However, issues with adaptability and traffic congestion in networks may make this strategy impractical for large-scale applications.

Aich et al. (2019) [38] and Rejeb et al. (2019) [22] provided insight into the revolutionary possibilities for blockchain technology in supply chain services. Supply chains might undergo a radical transformation thanks to this technology, which can also reduce fraud and increase transparency and traceability. Widespread adoption is still constrained by issues with overcoming integration concerns with current systems and guaranteeing compatibility. Alam (2019) [46] emphasized blockchain's crucial role on the Internet of Things. Blockchain technology has the potential to alter data communication and interaction amongst IoT devices by promoting data integrity, transparency, and decentralized control. Scalability problems and energy consumption continue to be key barriers to wider implementation. Pavithran (2020) [47] presented a blockchain framework designed for IoT setups. This strategy seeks to solve the distinct issues of data tampering and illegal access in IoT networks by improving data integrity and decentralized control. However, scalability problems and possible performance limitations must be carefully addressed during the installation process. Khrais (2020) [45] highlighted the potential advantages of combining IoT and blockchain in smart city development. This strategy has the potential to improve data security, efficiency, and enable novel services, resulting in the creation of sustainable and resilient urban infrastructure. However, integration issues and potential privacy problems must be carefully examined in order to fully realize the promise of this technology in smart city applications.

Shammar and Zahary (2021) [48] explored the security implications of combining blockchain with IoT. Their technique uses blockchain's immutable ledger and strong encryption to improve data security and reduce fraud risks in IoT networks. However, the implementation complexities and significant performance overhead require careful consideration. Hemalatha et al. (2021) [41] investigated the use of IoT and blockchain to monitor and secure healthcare data. This strategy guarantees immutable data records and increased security, which are critical for protecting patient privacy and preventing illegal access to sensitive medical information.

Alzuabi et al. (2022) [49] emphasized the significance of detecting and fixing any security flaws in these systems. Policymakers, industry leaders, and researchers must work together to develop successful frameworks that encourage innovation while limiting risks. Kumaresan et al. (2022) [43] and T. Wang et al. (2024) [42] presented techniques for addressing the scalability issues related with merging blockchain with IoT. These developments are critical for allowing large-scale deployments of the technology. Sallal et al. (2023) [51] and Magara & Zhou (2024) [52] addressed methods to include privacy-preserving mechanisms into blockchain-based IoT systems. This is critical in balancing the requirement for openness with security of information concerns, especially in highly sensitive sectors like healthcare.

Enhancement of security, data integrity, openness, and decreased fraud are recurrent benefits among the different techniques. Significant obstacles are, nonetheless, presented by difficulties with scalability, complexity of implementation, privacy, and possible performance cost. The many strategies and areas of concentration for combining blockchain with IoT are demonstrated in this thorough overview. All strategies have different advantages and confront different obstacles. Blockchain technology has a lot of potential to improve security, efficiency, and transparency in IoTsystems, but realizing its full potential in practical applications will require resolving challenges with scalability, interoperability, and law. For blockchain-based solutions to be adopted throughout IoT ecosystems, industry leaders, researchers, and legislators must work together to overcome these obstacles.

This article addresses the key problems of secure data management in the various sectors, especially in nuclear energy sector by exploring the integration of blockchain technology with IoT. In this study, we aim to investigate how this integration can improve data security, integrity, and privacy, which are of most important aspects in this domain. Our contributions to the field are as follows:

We provide a thorough overview of the integration of blockchain and IoT technologies, with a specific focus on the security and privacy concerns vital to nuclear energy applications. By recognizing limitations and prospects in integrating these technologies (IoT and Blockchain), our work extends significant insights for researchers and specialists in this sector. Additionally, we provided a flowchart that describes the key concerns involved in this integration, serving participants in envisioning the necessary elements of the process. Furthermore, we investigated possible solutions to the security and privacy challenges associated with integration of blockchain and IoT, advancing a basis for future research and development in this area. Our evaluation of blockchain's cryptographic transaction process improves interpretation of the security mechanisms involved, requiring technical insights into generally used algorithms and their functionality through pseudocode. Additionally, we also presented a secure data management framework exclusively intended for IoT applications, supported by a thorough block diagram. This framework introduces an overall solution for guaranteeing the security of data transmission and storage. By investigating these factors, our work adds to the existing research on using blockchain and IoT for safe data management in critical infrastructure applications such as nuclear energy.

## 3 Methodology

In light of integrating IoT and Blockchain technologies, this section explains the techniques and resources used to assess security and privacy issues as well as possible remedies. A comprehensive explanation of the methods used in our study may be found in the following subsections. In order strengthen our analysis, these subsections will contain thorough explanations, flowcharts, block diagrams, and mathematical formulas.

### 3.1 The potential of IoT and blockchain

As seen in Fig. 3, this section explores the potent synergy between blockchain and IoT technology. A new paradigm for data security and privacy is unlocked by the combination of blockchain technology and IoT across a number of industries, such as supply chain management, healthcare, and smart cities. This section explores the fundamental features of this potent synergy, emphasizing the advantages it provides in terms of security and privacy.

**Fig. 3:** Blockchain and IoT integration for enhanced data security and applications.

Based on several publications referenced in the literature review section, we developed a block diagram that illustrates how Blockchain and IoT are integrated for improved data security and other applications. This illustration demonstrates the way a variety of communication protocols, including as 6LoWPAN, LoRa, Bluetooth, ZigBee, and Wi-Fi, are used to connect IoT devices that are equipped with sensors and actuators to establish a strong IoT network. Through local processing of the data produced by these sensors, Edge artificial intelligence applications allow for anomaly detection, predictive maintenance, and real-time analytics. By employing consensus, hashing, and encryption techniques to verify transactions and record them irreversibly in a blockchain ledger, the integration with blockchain technology ensures the secure management of this data. The blockdiagram also emphasizes how important blockchain is to enabling particular applications where data security and integrity are crucial, like supply chain management, decentralized finance (DeFi), and healthcare data management. The illustration additionally demonstrates how technologically advanced blockchain abilities like privacy protections, scalability solutions, and smart contracts improve the overall security and functionality of the integrated system. With this block diagram, we present a thorough explanation of how the integration of IoT and Blockchain can result in secure, scalable, and effective data management in a number of essential sectors.

Table 2 summarizes current research (from 2022 to 2024) that investigate the integration of Blockchain technology with the IoT, concentrating on security, privacy, and data integrity. Each item represents separate research, complete with its own features and conclusions. Blockchain is commonly used in IoT contexts to improve security and decentralization, according to several research.

**Table 2:** Comprehensive review of blockchain integration in IoT for enhancing security, privacy, and data integrity.

References	Feature	Blockchain	IoT	Blockchain Security	Blockchain Application	Blockchain type	IoT application	IoT security	IoT privacy	IoT integrity	Solutions	IoT-Blockchain Integration
[55]	Blockchain-based IoT Device Security	✓	✓	Trust and authentication across IoT elements	Secure IoT device management, prevention of data breaches	Permissioned	IoT device management	✓	✗	✗	✓	✗
[54]	Location Privacy in IoT using LDP	✓	✓	Decentralized data storage, access control	Secure and private location data management	Permissioned	Smart homes, wearables, industrial monitoring	✓	✗	✗	✓	✓
[40]	Blockchain & IoT for Food Supply Chain	✓	✓	Enhanced traceability & tamper-proof records	Food Supply Chain	Permissioned	Farm-to-Fork Tracking, Smart Contracts for Transactions	✓	✓	✗	✓	✗
[53]	DeviceShadow-Blockchain for Secure IoT Data	✓	✓	Decentralized & tamper-proof shadow data storage	Enhanced data security & privacy	Permissioned	Focus on Shadow Data	✓	✗	✓	✗	✗
[60]	Integration of IoT with Blockchain	✓	✓	Secure IoT device management	secure control using blockchain and smart contracts	Permissioned	IoT device management	✓	✗	✗	✗	✓
[39]	Blockchain with IoT for Secure Manufacturing Supply Chain	✓	✓	Secure and tamper-proof transaction signing	Enhanced supply chain transparency & traceability	Permissioned	Manufacturing	✓	✗	✗	✗	✗
[57]	Blockchain for IoT security and privacy	✓	✓	Secure decentralization	✗	Public/Private	Smart objects	✓	✓	✗	✓	✓
[44]	Integration of IoT and blockchain with enhanced Security	✓	✓	Decentralized and tamper-proof system	✗	Public/Private, Consortium	Healthcare, smart cities, industrial automation	✓	✗	✓	✓	✓
[56]	Blockchain's Role in IoT Security	✓	✓	Immutable data records, auditable transactions	Secure data exchange, access control	Permissioned	Supply chain management, logistics tracking	✓	✗	✗	✗	✓
												
[58]	Edge Computing & Blockchain for Secure IoT	✓	✓	Secure data storage & processing at the edge	Improved security & privacy across the network	Permissioned	Healthcare, Agriculture, Manufacturing, Smart Cities	✓	✓	✗	✓	✓

While auditable transactions and tamper-proof records are popular aspects used in most studies to address data security, data privacy and integrity tend to receive less attention. To improve data security and integrity, almost all research use blockchain security in some way, such as decentralized storage or tamper-proof records. Items such as "Enhanced traceability & tamper-proof records" (Kaur et al., 2022) [40] and "Secure and tamper-proof transaction signing" (Madhwal et al., 2023) [39] clearly demonstrate this. Despite being less well-known, certain studies do discuss data privacy. For example, "DeviceShadow-Blockchain for Secure IoT Data" (Bao & Lu, 2022) [53] discusses better data privacy, while "Location Privacy in IoT using LDP" (He et al., 2022) [54]. addresses safeguarding location data.

The table covers a wide range of IoT applications where Blockchain integration is being explored. This includes supply chain management (Madhwal et al., 2023; Kaur et al., 2022) [39,40], healthcare (Velamakanni & Patwal, 2024) [44], and smart homes (He et al., 2022) [54]. According to the majority of research, permissioned blockchains—those with limited access—are the best option (Cp et al., 2022; Deepak et al., 2024) [55,56]. Studies by (Sinha, 2024) [57] and Velamakanni & Patwal (2024) [44], for example, place special emphasis on tamper-proof systems and safe decentralization, respectively, across a range of applications, from industrial automation to smart products and healthcare (Deepak et al., 2024). [56] emphasize that blockchain technology plays a crucial role in guaranteeing unchangeable data records and safe data sharing in supply chain management scenarios. The table presents many implementations of IoT applications, including edge computing for increased security (Nguyen et al., 2024) [58], traceability in food supply chains (Kaur et al., 2022), and secure location data management (He et al., 2022) [54]. These uses case highlight how flexible Blockchain may be in tackling certain IoT problems while maintaining data security and integrity.

A noteworthy finding from the table is the lack of focus that many research have paid to IoT privacy and Integrity. The majority of academics place greater emphasis on security and the related solutions than the privacy considerations, as seen by the fact that their Blockchain-based IoT solutions frequently lack specific privacy improvements. More effective privacy-preserving techniques may be the subject of future study in this field to supplement current security measures. Overall, although blockchain technology has the potential to improve data integrity and IoT security in a number of fields, there is still a great chance to better integrate and give privacy considerations top priority in these creative solutions.

#### 3.1.1 The significance of data preprocessing for security

The raw data that IoT devices gather is the first step towards safe and reliable data. On the other hand, inconsistencies and discrepancies may occur with this data. Analytical integrity may be jeopardized by outliers, or data items that differ noticeably from the average. Predictions drawn from incomplete data sets may also be incorrect. Multi-stage preprocessing is used to mitigate these weaknesses and guarantee data dependability and correctness. Using the Interquartile Range (IQR) to discover anomalies and deal with outliers is all part of this procedure. To guarantee a full data set for analysis, strategic approaches are also used to fill in the missing data points. Last but not least, the data is painstakingly cleaned out of noise and standardized to a standard scale. Data may be appropriately understood and analyzed thanks to this assurance of data integrity for later process steps [59].

#### 3.1.2 Effective encryption for enhanced security

After preprocessing, strong encryption protects the sensitive data. The illustration shows how to use two different key encryption methods, each with unique benefits. A public-private key pair is used for encryption and decryption in asymmetric encryption (RSA). Sensitive information is only accessible through the appropriate private key, which guarantees restricted access to data encrypted with the public key. A single shared key is used by symmetric encryption, Advanced Encryption Standard (AES) for both encryption and decryption. Its strong performance in encrypting substantial amounts of data within the system makes it appropriate for real-time data streams produced by IoT devices [61]. Additionally, digital signatures produced using private keys (ECDSA/EdDSA) are used. By confirming the veracity and integrity of the data, these signatures serve as a digital fingerprint and promote system confidence [62].

#### 3.1.3 The blockchain mechanism

The blockchain network is then updated with the pre-processed and encrypted data. This distributed ledger system provides a strong foundation for storing and validating transactions. The network uses consensus techniques like Proof of Work (PoW) and Proof of Stake (PoS) to carefully review and approve transactions. These transactions are permanently recorded on the blockchain when they are approved, guaranteeing their transparency and immutability [63]. In applications like supply chain management, where precise monitoring of product origins and authenticity verification are critical, this promotes confidence and security.

#### 3.1.4 Decryption and data integrity authentication

Depending on the encryption strategy used, data decryption is carried out using either symmetric (AES) or asymmetric (RSA) techniques after blockchain confirmation. The data has been encrypted and is now available for use and additional analysis inside the system. Data integrity must always be maintained. Data is assigned a unique fingerprint through the use of hashing algorithms, such the popular SHA-256 [59,63]. The hash value will vary in response to any unwanted data changes, making detection possible right away. In addition, identity validation and integrity checks serve as gatekeepers, guaranteeing the authenticity of data coming from IoTdevices and avoiding the introduction of unwanted data. The foundation of this security mechanism is made up of device signatures and verification using public key registries.

#### 3.1.5 Enhanced privacy with advanced cryptographic techniques

The figure presents sophisticated cryptographic approaches such as Attribute-Based Encryption (ABE), Homomorphic Encryption, and Zero-Knowledge Proofs (ZKPs) for cases where data privacy is critical, particularly in the healthcare and financial industries. These advanced instruments provide private data management while enabling secure data operations. Access control is made possible via attribute-based encryption, or ABE. This makes sure that only people who are allowed and have the right qualities may access the info that is meant for them. This relates to patient privacy in healthcare applications since patient data is only accessible by authorized medical staff. Similar to this, it protects financial security in banking applications by limiting access to financial information [1,64]. Computations on encrypted data can be completed without first requiring decryption thanks to homomorphic encryption. This allows for useful analytics while maintaining data privacy. For instance, it enables the study of medical data in the healthcare industry without disclosing the personal information of individual patients. ZKPs enable users to demonstrate their ownership of certain data (such as service eligibility) without disclosing the data itself. This further protects the privacy of users. For example, consumers can verify they are eligible for a service without disclosing personal information.

### 3.2 Framework for data flow and IoT applications

Fig. 4 explores the specifics of the Internet of Things' application and data flow structure, which has impacted a number of sectors. Secure connectivity and centralized data management via an IoT hub are crucial, and this paradigm emphasizes their importance.

**Fig. 4:** Data flow framework for secure IoT applications with centralized management.

#### 3.2.1 A diversity of applications from various disciplines

The diagram reveals an intricate web of IoT applications produced through numerous fields. Intelligent solutions that optimize energy distribution (smart grid management), minimize usage (energy consumption optimization), and continuously monitor the environment (environmental monitoring) to guarantee sustainability are all beneficial to smart surroundings. IoT-enabled smart cities use upgraded surveillance systems (Security Systems), smart houses for improved convenience and security, and better traffic flow (Traffic Management). Predictive maintenance technologies reduce equipment downtime, real-time asset tracking enables proactive maintenance, and simplified automation guarantees effective production processes in the industrial sector (Industrial Automation). Wearable health trackers that measure a person's vital signs and remote patient monitoring systems that enable medical professionals to check a patient's health from a distance are examples of smart living applications [65,66]. Robust fraud detection technologies and secure payment systems are advantageous for financial services. Lastly, fleet management systems and linked car diagnostics are employed in the smart mobility arena to provide real-time vehicle health monitoring and optimal operations. Although these apps provide many advantages, there are security risks as well. Sensitive data gathered from sensors and devices may be altered or accessed without authorization, which might have dangerous repercussions. In order to guarantee data security and privacy throughout the whole data flow process, the framework must handle these issues.

#### 3.2.2 A methodical approach to data acquisition and preprocessing

The preparation and acquiring of the data produced by these many applications are done in an organized manner. The workhorses of data gathering, sensors and actuators, are strategically placed across a range of applications to get pertinent data. Then, this data is safely transferred via reliable connectivity options that guarantee effective data transfer. In order to control the data flow between sensors and actuators and the larger network, gateways serve as intermediate devices. These gateways combine data from many sources and get it ready for additional processing. Secure communication for the transfer of this data is made possible via the LoRa/6G Network, a low-power, wide-area network [62,67]. The Data Collection & Preprocessing step next entails painstakingly compiling and getting the gathered data ready so that it can be easily analyzed and formatted correctly.

#### 3.2.3 The IoT hub

The IoT Hub serves as a hub for data from many applications, making it the brains of the whole system. To enable centralized control, all of the preprocessed data is directed via the IoT hub. This place places a high priority on security, and the hub protects communications and data transactions from potential breaches and illegal access. Strong security protocols are put in place to protect the confidentiality and integrity of data [52,68]. In order to safeguard data during transmission and guarantee that sensitive information is not compromised, secure communication procedures are also enforced across the network.

#### 3.2.4 Instructions and data processing

After data arrives to the IoT hub, it is processed once again to produce useful insights and orders. To extract useful information that can guide decision-making processes, data from apps is carefully examined. This analysis is used to develop particular instructions that direct the behavior of different systems and devices in the network. For the full framework to be implemented with automatic replies and changes, these instructions are essential [63,69]. Additionally, the framework makes it easier for users to engage with one another. It enables administrators and end users to get insights, manage programs as needed, and issue instructions based on data processing. Users are empowered to make well-informed decisions by the insights obtained from data analysis. Furthermore, actuators—the physical equivalents of commands—receive instructions derived from the processed data and execute the required actions, completing the circle from data gathering to real-world application.

#### 3.2.5 Secure communication

Throughout the whole framework, there is emphasis on the value of secure communication. Secure communication channels are essential for data transmission over gateways and networks, centralized processing in the IoT hub, and initial data acquiring by sensors and actuators. This strong security framework protects availability, confidentiality, and integrity of data, preventing illegal access and guaranteeing the dependable functioning of IoT devices [59,70]. The usefulness and trustworthiness of the IoT ecosystem are largely dependent on the security measures put in place at every point of the data flow. A detailed description of the data flow structure and the intricate operations of IoT applications may be found in Fig. 5. The statement emphasizes the interconnectedness of diverse applications across many areas and the crucial role that security plays in ensuring the dependable and effective functioning of connected devices. Utilizing the enormous potential of IoT while reducing the related security risks is made possible by this architecture.

**Fig. 5:** Multi-step secure data management framework for IoT leveraging algorithms and blockchain.

### 3.3 Secure data management framework

An effective data management system is essential to the safe and effective functioning of IoT applications. This section examines a thorough architecture created to safeguard confidentiality, privacy, and data integrity inside the IoT ecosystem [43]. It describes a multi-step procedure that takes into account frequently used algorithms for both IoT and blockchain technologies, as well as data pretreatment, encryption, blockchain integration, and state-of-the-art security approaches.

#### 3.3.1 Data preprocessing & encryption

Raw data is the first step in the data preprocessing and encryption process, during which it is transformed in a number of ways to get ready for safe transmission and storage. IQR is the first technique used to identify and manage outliers. Next, in order to guarantee that the data set is full, any missing values are imputed. After that, the data is standardized to a specified range, which improves consistency and dependability. Following these procedures, the data is formatted and cleaned, preparing it for encryption [50]. This is where the decision is made between symmetric encryption with AES and asymmetric encryption with RSA. The data is encrypted using a shared AES key in symmetric encryption. On the other hand, asymmetric encryption uses a private key signature to verify the validity of the data using methods like EdDSA or ECDSA. Encrypted data that is safe for transmission or storage is the end product of these procedures.

#### 3.3.2 Blockchain network verification

The procedure for verifying and appending transactions to the blockchain is described in the section on Blockchain Network Verification. PoW or PoS are the two options available for transaction validation after a transaction is broadcast to the network [17,69]. Whereas PoS depends on validators verifying the transaction based on their stake in the network, PoW requires miners to solve a challenging mathematical problem using the SHA-256 algorithm. The legitimacy of the transaction is then assessed by the network. The transaction is declined if it is found to be invalid. If it is legitimate, it gets put to the blockchain after going through additional verification (in the case of proof-of-stake). In order to preserve the network's integrity and security, this procedure makes sure that only verified transactions are added to the blockchain.

#### 3.3.3 Data decryption

Encrypted data is transformed back into its original format for usage during the data decryption stage. Depending on whether symmetric (AES) or asymmetric (RSA) encryption was previously employed, the proper decryption technique is selected. The data is decrypted using the shared AES key in symmetric decryption. Asymmetric decryption, on the other hand, uses the private RSA key. This stage makes sure that the decrypted data is available and prepared for additional processing or analysis while upholding the information's confidentiality and integrity.

#### 3.3.4 Integrity verification & device authentication

Device and integrity verification for data and devices to be valid and intact, authentication is essential. First, the device generates a signature, which is then checked against a public key registry [71]. To verify that the data is valid, the public key is utilized. The data is confirmed and authenticated if the signature can be independently checked. If the verification is unsuccessful, though, it suggests an integrity or authentication problem. Ensuring the authenticity and integrity of data is crucial in preventing tampering or unauthorized access. This step protects against such risks.

#### 3.3.5 Secure communication channel establishment

To create a secure connection, this procedure begins with a Transport Layer Security (TLS) handshake. The server delivers its certificate for validation; it is usually a component of the blockchain network. Next, Public Key Infrastructure is used to verify this server certificate (PKI). The construction of a secure connection is hindered if the certificate verification process is unsuccessful, and an error is reported. Secure data transfer is made possible by the establishment of a secure TLS connection following successful verification. By doing this, you can be confident that no data is ever intercepted or tampered with during transmission between the client and server.

#### 3.3.6 Data decryption & integrity check

This step makes sure the decrypted data stays whole and unchanged. First, the original data's hash is kept. The SHA-256 technique is used to determine the data's hash once it has been decrypted. Next, the computed hash and the stored hash are contrasted. The integrity of the data is verified if the hashes match. In the event that the hashes do not match, an error will occur as it suggests that the data has been altered. Maintaining the data's dependability and trustworthiness requires taking this vital step to ensure that it hasn't been changed throughout transmission or storage.

#### 3.3.7 Privacy preserving techniques

Privacy-preserving methods may be included into the data management framework to improve security and user control over their data even further. Beyond standard encryption, these methods provide more precise access control and data processing capabilities without jeopardizing secrecy. Only authorized users can access encrypted data thanks to ABE, which encrypts data based on particular user behaviour. Homomorphic encryption protects privacy during analysis by allowing calculations to be performed directly on encrypted data. Finally, individuals may demonstrate their possession of certain data without disclosing it thanks to ZKPs. In order to approve processing, the blockchain network checks these proofs [59,63]. Homomorphic Encryption enables computations directly on encrypted data, ensuring privacy during analysis. Finally, ZKPs allow users to prove they possess certain data without revealing it. Through the implementation of these strategies, the framework may guarantee the confidentiality of data throughout its entire lifespan and confer additional authority to users, therefore cultivating a more secure and privacy-preserving environment for nuclear energy applications.

To further improve security and operational efficiency, it will be essential for practical evaluation to include real-world data from nuclear plants into testbeds and simulations and to look into deep learning models for anomaly detection and predictive maintenance [63,69]. By tackling these issues, scientists and programmers may build a strong, safe, and expandable framework that promotes a more dependable and safe nuclear energy infrastructure, eventually opening the door for its actual use in nuclear power plants.

### 3.4 Blockchain-IoT integration's security and privacy challenges

There are a lot of security issues with integrating blockchain with IoT, and these issues might seriously affect the system's dependability. Fig. 6 is the block diagram that shows how security issues and privacy concerns are addressed through focused solutions. Encryption, ACLs, RBAC, and differential privacy strategies are some of the particular solutions linked to each security problem, including Sybil attacks, data breaches, and flaws in consensus mechanisms. Strengthened security measures and privacy-preserving approaches are also implemented to address privacy issues, such as user identity disclosure, data tracking, and potential abuse [9,[72], [73], [74], [75]].

**Fig. 6:** Mitigating security challenges and privacy concerns in Blockchain-IoT integration.

#### 3.4.1 Blockchain-IoT integration security challenges

To maintain the network's resilience and dependability, a number of significant security issues posed by the integration of blockchain technology with IoT devices must be addressed.

• ***Sybil attacks:*** These kinds of attacks require a malicious attacker establishing many fraudulent identities. In particular, for operations that call on consensus mechanisms like voting and transaction validations, this might overload the network and cause resource exhaustion. These fraudulent identities have the ability to negatively affect performance, interfere with regular network operations, and even provide an attacker the ability to control network activity [75].
• ***Data breaches on IoT devices:*** Because of their susceptibility to malware and insufficient authentication procedures, IoT devices are frequently the target of data breaches. Data loss, manipulation, or theft may result from weak authentication, which gives unauthorized users access to the network. Threats to the network as a whole might arise from malware that further tampers with the integrity of the data that IoT devices gather and analyze [74].
• ***Consensus mechanism weaknesses***: Blockchain depends on consensus methods to approve transactions and preserve the ledger's integrity. These systems may, nonetheless, be susceptible to weaknesses. For instance, 51 % attacks, in which a single party with more than half of the network's mining capacity manipulates the blockchain, can affect PoW systems. This might undermine the system's credibility by encouraging double-spending and other illegal behavior [73].

#### 3.4.2 Blockchain-IoT integration privacy considerations

The intrinsic transparency and immutability of blockchain technology make privacy a significant problem in the context of blockchain-IoT integration [72].

• ***User identity exposure:*** Transaction data on blockchain is open to the public due to its openness. User identities may be revealed if public keys are connected to real-world identities. This connection may jeopardize user privacy by disclosing private information such as transaction history and behavioral patterns.
• ***Data tracking:*** IoT devices gather enormous volumes of data, some of which may contain private data. Without the user's permission, this data may unintentionally be gathered, saved, and monitored. Because malevolent parties may use the information for evil intent, unauthorized access to this data may result in serious privacy violations.
• ***Potential for misuse***: Among the main concerns is the potential for data misuse. Private rights might be violated by data modification and unapproved data exchange. Using IoT data modification and illegal sharing of private information to trick or deceive people are examples of this. Regarding personal privacy and system confidence, these acts may have negative effects.

#### 3.4.3 Security and privacy solutions

A variety of security and privacy techniques may be used to minimize these issues, assuring the secure and effective operation of blockchain-IoT systems [72,75].

• ***Secure data storage:*** Both in transit and at rest, data must be encrypted. Unauthorized individuals cannot access or read data that has been encrypted. By limiting who has access to particular network resources, Access Control Lists (ACLs) improve security even more by making sure that only authorized users may handle sensitive data.
• ***Access control mechanisms:*** Users can only access the data required for their responsibilities by using Role-based Access Control (RBAC), which limits system access based on user roles. By confirming the identification of users and devices, identity management systems—especially those built on Public Key Infrastructure (PKI)—allow safe network communication.
• Differential privacy techniques: These methods encrypt data before sharing it in order to safeguard certain data points. This data disturbance permits valuable aggregate data analysis while guaranteeing the privacy of individuals. Aggregate reporting further improves privacy by combining data from many different sources to offer insights without disclosing specific data points.

A thorough framework is created by comprehending and resolving the unique security and privacy issues with these solutions. This guarantees the security, dependability, and ability to preserve user privacy of blockchain-IoT systems while preserving effective and transparent operations. In order to successfully integrate blockchain and IoT technologies, researchers, industry stakeholders, and legislators must work together to create and implement these solutions [76].

Table 3 explores the impact of addressing various security and privacy challenges faced in Blockchain-IoT integration. It details potential performance and scalability implications, along with key considerations for implementation. This table delineates the security and efficiency challenges inherent in integrating blockchain and IoT technologies, offering potential solutions and implementation considerations. Addressing Sybil Attacks, which involve fake identity creation to disrupt networks, may involve adopting PoS or reputation-based systems, albeit with added validation overhead. Meanwhile, countering Data Breaches on IoT Devices necessitates robust authentication, secure boot procedures, and encryption, albeit with potential processing overhead on resource-limited devices. Consensus Mechanism Weaknesses, such as vulnerabilities in PoW, may require transitioning to PoS or BFT mechanisms, balancing security with scalability considerations. User Identity Exposure risks from public ledgers can be mitigated with techniques like ring signatures or zero-knowledge proofs, albeit with increased verification complexity. Data Tracking challenges, involving inadvertent collection and unauthorized access, can be addressed with fine-grained access control and data aggregation, though may increase processing demands for data anonymization. Finally, tackling the Potential for Misuse, such as data manipulation or misuse, may necessitate secure data storage, access controls, and governance policies, albeit with added complexity for data management within the ecosystem.

**Table 3:** Balancing security and efficiency impact and considerations of addressing blockchain-IoT challenges.

Security/Privacy challenge	Description	Potential solutions	Impact on performance/scalability	Considerations for implementation
Sybil attacks	Infiltrators create fake identities to disrupt the network.	PoS, Reputation-based systems	May introduce additional validation overhead.	Requires careful design of reputation scoring mechanisms to prevent manipulation.
Data breaches on IoT devices	Weak authentication and malware infections on resource-constrained devices expose data.	Strong authentication, Secure boot, Firmware updates, Data encryption	Increased processing requirements for encryption/decryption on IoT devices.	Lightweight encryption algorithms and secure boot procedures optimized for resource-constrained devices.
Consensus mechanism weaknesses	Certain mechanisms like PoW are vulnerable to 51 % attacks.	PoS, Byzantine Fault Tolerance (BFT)	Complexity of implementation for BFT can impact scalability.	Choosing a consensus mechanism that balances security with efficiency based on the application's needs.
User identity exposure	Public ledgers can reveal user identities.	Ring signatures, Zero-knowledge proofs, Consortium blockchains	Increased complexity for transaction verification.	Requires careful integration with existing identity management systems.
Data tracking	Inadvertent collection and unauthorized access compromise privacy.	Fine-grained access control, Data aggregation, Differential privacy	May introduce additional processing overhead for data anonymization.	Balancing data utility with privacy needs through user-centric control mechanisms.
Potential for misuse	Malicious actors might manipulate data or misuse user information.	Secure data storage, Access control mechanisms, Data governance policies, Regulations	Increased complexity for data access management.	Establishing clear ownership and responsibility for data within the Blockchain-IoT ecosystem.

### 3.5 Cryptographic secure transaction process in blockchain

The cryptographic secure transaction process is a fundamental aspect of blockchain technology, especially when considering security and privacy. This section delves into the details of how data transmission within a blockchain network is secured through cryptography. We reviewed at the particular phases in this process and offered a road map for comprehending how blockchain transactions preserve the authenticity, secrecy, and integrity of data.

#### 3.5.1 Symmetric data encryption

The foundation for protecting private data in blockchain transactions is symmetric encryption. Using a shared secret key $K_{s}$ and an encryption technique like AES, this approach transforms the original information (D) into a format that is incomprehensible $E_{D}$. This key is held by both the sender and the recipient, allowing users to encrypt and decrypt the information, respectively, protecting secrecy while being sent via possibly unsafe networks [76]. equation (1) represents symmetric data encryption.

(1) $$E_{D}=E_{s}\left(D,K_{s}\right)$$

Here, $E_{D}$ represents the encrypted data generated by applying the symmetric encryption function $E_{s}$ to the original data (D) using the secret key $K_{s}$. This encrypted form safeguards data confidentiality, thwarting unauthorized access even if intercepted within the blockchain network. However, secure sharing of the secret key is paramount. If compromised, access to the key could lead to decryption of the data by unauthorized parties.

#### 3.5.2 Asymmetric key encryption

Building on symmetric encryption, asymmetric encryption is essential for secure blockchain transactions. Unlike symmetric encryption, which uses a single shared key, asymmetric encryption employs a key pair a public key and a private key [77,78]. In blockchain, this involves encrypting the symmetric key $K_{s}$ with the recipient's public key $K_{pub}$. equation (2) illustrates this process:

(2) $$E_{K_{s}}=E_{a}\left(K_{s},K_{pub}\right)$$

Here, $E_{a}$ is the asymmetric encryption function. $K_{s}$ is the symmetric key to be encrypted, and $K_{pub}$ is the recipient's public key. The resulting $E_{K_{s}}$ represents the encrypted symmetric key, ready for transmission over potentially insecure channels. Leveraging asymmetric encryption enables secure communication within blockchain's decentralized environment, reducing risks associated with key exchange and interception.

#### 3.5.3 Data hashing and timestamp addition

After encryption in a blockchain transaction, data hashing generates unique identifiers, ensuring data integrity. Applying a hash function (H) to the encrypted data $E_{D}$ produces a fixed-size digest known as the hash value $H_{D}$. This fingerprint represents the content uniquely. Any alteration to $E_{D}$ results in a different $H_{D}$, exposing tampering attempts. Presented by equation (3):

(3) $$H_{D}=H\left(E_{D}\right)$$

Through data hashing, organizations secure communication channels in blockchain, mitigating risks of tampering and ensuring data transaction reliability [77,79]. In secure blockchain transactions, incorporating a timestamp enhances the integrity and immutability of transmitted information. After generating the hash value $H_{D}$ for the encrypted data, a timestamp (T) is strategically integrated into the hashing process. This digital time stamp marks the exact transaction moment. Equation (4) represents this process:

(4) $$H_{D,T}=H\left(C\left(H_{D},T\right)\right)$$

Here, C denotes the concatenation operation merging the timestamp with the hash value. The resulting composite hash ($H_{D},T$) encapsulates both data content and transaction time, strengthening data security. Any attempt to alter data or timestamp produces a different hash value, revealing tampering. This timestamp also enhances transaction history verifiability, fostering transparency in the blockchain network.

#### 3.5.4 Digital signature and message formation

In blockchain's cryptographic secure transaction process, digital signatures ensure authenticity, integrity, and non-repudiation of transmitted information. After creating the composite hash ($H_{D,T}$) containing encrypted data and timestamp, the next step involves digitally signing this hash value [80,81]. Using the sender's private key ($K_{priv}$), a unique cryptographic seal for the transaction is generated. Equation (5) illustrates this process:

(5) $$Sig_{D}=Sig\left(H_{D,T},K_{priv}\right)$$

Here, Sig represents the digital signature generation function. $H_{D,T}$ represents the composite hash value, and $K_{priv}$ signifies the sender's private key. Digital signatures authenticate the sender's identity using the corresponding public key ($K_{pub}$) and ensure data integrity. Any alterations to the data invalidate the signature. Digital signatures also ensure non-repudiation, enhancing accountability and reliability in communication.

In the domain of secure data transmission within blockchain networks, message formation holds significant importance. This critical step involves constructing a comprehensive message (M) that encapsulates all essential components necessary to guarantee the integrity, authenticity, and confidentiality of transmitted information. The message (M) encompasses several crucial elements, including the encrypted data itself ($E_{D}$), the encrypted symmetric key ($E_{K_{s}}$) used for decryption, the composite hash value incorporating the timestamp ($H_{D,T}$) for data integrity verification, and the digital signature ($Sig_{D}$) for sender authentication [82]. This message formation process is succinctly represented by equation (6):

(6) $$M=\left(E_{D},E_{K_{s}},H_{D,T},Sig_{D}\right)$$

Here, M constitutes a tuple comprising the encrypted data, encrypted symmetric key, composite hash with timestamp, and digital signature. By amalgamating these components into a unified message, organizations ensure that all requisite information for secure communication is effectively conveyed.

#### 3.5.5 Blockchain consensus mechanisms

***Proof of work (PoW):*** In blockchain technology, PoW is a fundamental consensus mechanism ensuring the security and immutability of the distributed ledger. Miners aim to discover a nonce (N) combined with the block header (B) yielding a hash value below a target threshold (T), validating and appending new blocks to the blockchain. Equation (7) illustrates the PoW mechanism:

(7) N=min{n:H(B‖N)<T}

Here, (B) represents the block header, and (H) denotes the hash function applied to their concatenation. Miners show computational effort to protect the network by repeatedly searching for an appropriate nonce [81,83]. The difficulty of finding a valid nonce adjusts based on the target threshold, enhancing blockchain security against tampering. Though PoW ensures reliability and tamper-resistance, newer consensus mechanisms offer alternative approaches for transaction validation. A full understanding of the mechanisms behind the PoW process is provided by Algorithm 1's detailed pseudocode description, which explores the process's many complexities.

Algorithm 1 Pseudo-code for PoW

**Table:** 

**Input:** T, P, A (Transaction data, PrevHash, AdditionalData) **Output:** B (Mined block) **Initialize:** N = 0 (Initialize nonce) candidateBlock = null **for** t = 0 to T-1 do $Block_{candidate}$ = $Block_{generate}($ T, P, N, A) **if** isValidProof($Block_{candidate}$) then **return**$Block_{candidate}$ **else** **return** N = N + 1 **end** **end** **return** B

Algorithm 2 Pseudo-code for PoS

**Table:** 

**Input:** B, A (Current block data, List of authorized validators) **Output:** B' (Valid block with valid proof) **for** each a ∈ A do: $S_{a}$ = getStake(a) $S_{total}$ = sum($S_{a}$ for a ∈ A) P(a) = $S_{a}$/$S_{total}$ v = selectValidator(A, P) **while** (True): B' = createBlock(v, B) **if** (isValidProof(B′, v)) then **return** B′ **end** **return** None

***Proof of stake (PoS):*** Under PoS, a validator selection mechanism is used to create and validate new blocks on a network. PoS takes advantage of a validator's bitcoin holdings, as opposed to PoW, which employs processing power. This staked cryptocurrency acts as collateral, and validators with a larger stake have a higher probability of being chosen to participate in the consensus process [81,84]. The selection probability for a validator, denoted by P(a), is directly proportional to its stake ($S_{a}$). This means validators with a significant financial investment in the network (represented by their stake) are more likely to be chosen. This relationship is mathematically expressed in equation (8).

(8) $$P\left(a\right)=\frac{S_{a}}{S_{total}}$$

This economic incentive structure in PoS encourages validators to act honestly. Because their stake is at risk, validators are highly motivated to follow the network's rules and contribute to its security. Additionally, PoS offers a significant advantage over PoW in terms of energy consumption. By eliminating the need for computationally intensive tasks like solving complex puzzles, PoS blockchains can operate with much lower energy requirements, making them a more sustainable choice. For a more thorough understanding of the PoS selection process, Algorithm 2 provides the pseudocode outlining the steps involved in validator selection.

***Delegated proof of stake (DPoS):*** DPoS builds upon the foundation of PoS by introducing a democratic voting system. In a DPoS blockchain, token holders don't directly participate in block validation. Instead, they elect a limited set of delegates (witnesses or block producers) to represent them in the consensus process. These delegates are responsible for creating and validating new blocks [62,76]. Similar to PoS, the probability of a validator (a) being selected (P(a)) is influenced by their stake ($S_{a}$). However, DPoS introduces an additional factor: voting weight ($W_{a}$). This weight reflects the collective stake of token holders who have voted for that particular delegate. equation (9) captures this combined influence:

(9) $$P\left(a\right)=\frac{S_{a}+W_{a}}{S_{total}+W_{total}}$$

DPoS offers several advantages over PoS. By concentrating validation power in a smaller set of elected delegates, DPoS achieves greater scalability and transaction processing efficiency. Additionally, it allows for a more distributed form of participation. Token holders can indirectly contribute to securing the network by voting for delegates they trust. This distributed voting process reduces the computational burden on individual token holders compared to direct PoS participation. In Algorithm 3, we've provided the pseudocode to offer a more comprehensive insight into the delegate selection process of Delegated Proof of Stake (DPoS).

Algorithm 3 Pseudo-code for Delegated Proof of Stake (DPoS)

**Table:** 

**Input:** B, $S_{v}$ , T (Current block data, Stake of the current node, Threshold) **Output:** B' (Valid block with valid proof) D = getDelegatesByVote(B) **for** each d in D: **if** (d = = current_node): weighting:=S_v/total_stake(B) **if** (T !=None and S_v < T): **continue;** B':=createBlock(d, weighting) **if** (isValidProof(B′, d)) then **return** B′ **end** **end** **return** None

***Byzantine fault tolerance (BFT):*** BFT is a consensus algorithm designed to achieve agreement in a distributed system even if some nodes exhibit Byzantine failures. These failures can encompass crashes, omission of messages, or even malicious actions where nodes deliberately send misleading information. BFT protocols establish communication channels and message exchange patterns among nodes to reach consensus on the validity of transactions and the current state of the network. BFT uses a mix of message exchange and agreement rules to reach consensus, in contrast to PoS and Delegated Proof of Stake (DPoS), which depend on financial incentives. In permissioned blockchain systems, where users are pre-identified and trusted, this approach is frequently employed. The scalability of BFT protocols may be impacted by the fact that, in comparison to other consensus techniques, they may need a greater number of message exchanges [79,85]. Algorithm 4 provides pseudocode describing general stages that BFT protocols might take to reach agreement, providing a more thorough understanding of the mechanisms involved in BFT.

Algorithm 4 Pseudo-code for BFT consensus algorithm

**Table:** 

**Input:** V, M, f (Set of validators, Proposed message/block to be agreed upon, Maximum number of faulty validators) Output: C (Consensus decision on the message/block M) **Initialize:** quorum = |V| - f **#Propose Phase:** leader:= selectLeader(V) leader.broadcast(M) **#Prepare Phase:** **for** each validator vi in V do **if** isValidMessage(M) then vi.send(prepare, M) to all validators//Send prepare message **end** **end** **#Commit Phase:** for each validator vi in V do if receive (prepare, M) vi.send end end **#Decision Phase:** for each validator vi in V do if receive (commit, M) return C = M **end** **end** **end** **return** None

#### 3.5.6 Adding and verification blockchain

Appending to the blockchain is essential for ensuring integrity, transparency, and security at the end of a blockchain transaction. A new block is added to the blockchain after the transaction message (M) and associated nonce (N) have been produced and verified. Equation (10), which depicts this process:

(10) B∪(M,N)

The blockchain is represented by B, and the tuple ((M, N)) is added to it using the union operator (⊎). This method keeps the network's transaction order and integrity intact, since each confirmed transactions become parts of the blockchain's record. Leveraging blockchain's immutability, organizations ensure trustworthiness of transactional data, enhancing transparency and accountability [81,86]. Immutability also bolsters blockchain security, as altering a past transaction would require modifying all subsequent blocks, which is computationally infeasible. Following the appending of a transaction to the blockchain, blockchain verification ensures the network's integrity. Participants collectively verify the added transaction's legitimacy by confirming its digital signature ($Sig_{D}$) using the sender's publicly known key ($K_{pub}$). Equation (11) illustrates this process:

(11) $$Verify\left(Sig_{D},H_{D,T},K_{pub}\right)=True$$

Here, the verification function assesses if the digital signature matches the hashed data, incorporating both the encrypted data and timestamp, using the sender's public key. This gatekeeping step ensures that only authorized parties with the corresponding private key can create valid transactions for the blockchain.

#### 3.5.7 Symmetric key and data decryption

Upon successful verification of a transaction, the next step involves decrypting the encrypted symmetric key ($E_{Ks}$)) to retrieve the original symmetric key ($K_{s}$) used for encrypting the transaction data. This decryption is essential for accessing the original plaintext information. Equation (12) represents this process:

(12) $$K_{s}=E_{a}^{-1}\left(E_{Ks},K_{priv}\right)$$

Here, $\left(E_{a}^{-1}\right)$ denotes the inverse function of the asymmetric encryption process. The original symmetric key $K_{s}$ is obtained by decrypting the encrypted symmetric key $E_{Ks}$ using a private key $K_{priv}$. Network users now have access to the encryption key required to unlock private transaction data thanks to this decryption step. The secrecy of transactional data is maintained throughout its lifespan in blockchain networks by secure key management [82]. Once the symmetric key $K_{s}$ has been successfully decrypted, the encrypted data $E_{D}$ must be decrypted in order to recover the original, legible data. Authorized users can see and use the information regarding the transaction in its original state for processing, analysis, or archiving thanks to this decryption procedure. This procedure is represented by equation (13):

(13) $$D=E_{s}^{-1}\left(E_{D},K_{s}\right)$$

This indicates that the symmetric encryption process's inverse function is represented by $E_{s}^{-1}$. To recover the original plaintext data (D), the encrypted data is decrypted using the decrypted symmetric key. In order to maintain the security and integrity of information related to transactions throughout its lifetime, safe key management is crucial inside blockchain networks, as this decryption phase emphasizes.

#### 3.5.8 Data integrity check

Reliability and trust are essential components of a blockchain network, and they must be preserved. In order to ensure the legitimacy of decrypted data, the data integrity verification phase confirms that the data has not changed after encryption [81]. In this procedure, the hash of the decrypted data $E_{D}$ is recalculated utilizing the primary hash function H, and the hash $H_{D}$ is compared to it. This integrity check validation is seen in Equation (14):

(14) $$H\left(E_{D}\right)=H_{D}$$

The hash of the decrypted data is shown above as $H\left(E_{D}\right)$, whereas $H_{D}$ stands for the original hash that was acquired during data hashing. Data integrity is verified by matching hashes, which reassure users of the data's original condition. The immutability and validity of transactional data inside the blockchain network are strengthened by this crucial phase, which also helps to avoid data tampering or illegal adjustments.

Table 4 lists the sequential procedures needed for cryptographic process of transactions in blockchain networks, along with an explanation and the equations that relate to each procedure. The operations listed above, which include hashing, encryption, data verification, consensus techniques, and signature generation, improve the security and integrity of transactions inside the blockchain network.

**Table 4:** Steps in cryptographic transaction processing within blockchain networks.

Step	Description	Equation
Symmetric data encryption	Encrypt data (D) with symmetric key ($K_{s}$)	$E_{D}=E_{s}\left(D,K_{s}\right)$
Asymmetric Key encryption	Encrypt symmetric key ($K_{s}$) with public key ($K_{pub}$)	$E_{K_{s}}=E_{a}\left(K_{s},K_{pub}\right)$
Data hashing	Generate hash ($H_{D}$) of encrypted data ($E_{D}$)	$H_{D}=H\left(E_{D}\right)$
Timestamp addition	Add timestamp (T) to the hash ($H_{D}$)	$H_{D,T}=H\left(C\left(H_{D},T\right)\right)$
Digital signature	Sign hashed data ($H_{D,T}\})$ with private key ($K_{priv})$	$Sig_{D}=Sig\left(H_{D,T},K_{priv}\right)$
Message formation	Form message (M) with encrypted data, encrypted key, hash, timestamp, and signature	$M=\left(E_{D},E_{K_{s}},H_{D,T},Sig_{D}\right)$
PoW	Find nonce (N) satisfying PoW requirement	N=min{n:H(B‖N)<T}
PoS	Select validator based on stake ($S_{a}$)	$P\left(a\right)=\frac{S_{a}}{S_{total}}$
DPoS	Select validator based on stake ($S_{a}$) and voting weight ($W_{a}$)	$P\left(a\right)=\frac{S_{a}+W_{a}}{S_{total}+W_{total}}$
BFT	Consensus among validators based on voting	$f=\lceil \frac{2}{3}n\rceil -1$
Appending to blockchain	Append message (M) and nonce (N) to blockchain (B)	B←B∪(M,N)
Blockchain verification	Verify signature using public key ($K_{pub}$)	$Verify\left(Sig_{D},H_{D,T},K_{p}ub\right)=True$
Symmetric key decryption	Decrypt symmetric key ($K_{s}$) with blockchain's private key ($K_{\text{priv}})$	$K_{s}=E_{a}^{-}1\left(E_{K_{s}},K_{priv}\right)$
Data decryption	Decrypt data (D) using decrypted key ($K_{s}$)	$D=E_{s}^{-}1\left(E_{D},K_{s}\right)$
Data integrity check	Recompute hash of encrypted data ($E_{D}$) and compare with original hash ($H_{D}$)	$H\left(E_{D}\right)=H_{D}$

## 4 Blockchain technology in nuclear energy

Fig. 7 depicts a thorough flowchart of blockchain technology's incorporation into the nuclear energy business. The goal is to accomplish improved productivity, reliability, safety, and sustainability. The flowchart underlines the need of assessing the efficacy of each implementation stage before moving on to the next.

**Fig. 7:** Enhancing nuclear energy with a flowchart for integrating blockchain technology.

### 4.1 Supply chain management

Supply chain management optimization is the primary step of blockchain's initial use in the nuclear energy field. To determine what needs to be improved, a comprehensive assessment is carried out first. Considerations included in this assessment include the potential advantages of implementing a blockchain solution, any hazards connected with the present framework, and inefficiencies that already exist. A system based on blockchain technology is put into place if the assessment finds that a more effective supply chain is required. In order to verify nuclear materials' legitimacy and stop their spread, this system painstakingly records their origin and movement along the supply chain. The goal of the implementation is to provide a visible and safe record of every movement and transaction that occurs inside the supply chain. The new system's efficacy is evaluated once it is put into place. Measuring cost savings, improved security, and transparency are the main objectives of this evaluation. If the supply chain management using blockchain technology works, the process moves on to the next phase, which is asset management.

### 4.2 Asset management

The physical infrastructure for nuclear energy is the subject of asset management in the second stage. The first step in this process is to assess if improved asset management techniques are necessary. An assessment of asset management's existing situation is conducted in order to identify instances in which the application of blockchain technology could improve operations. An asset management system built on blockchain is put into place if the necessity is determined. The goal of this system is to capture detailed information on asset ownership, scheduled maintenance, and regulatory compliance. The system seeks to increase the openness and efficiency of managing nuclear assets by utilizing blockchain technology. All data is guaranteed to be precise, unchangeable, and readily available because to blockchain's data management features. Next, the affordability, efficiency of operation, and accessibility improvements of the blockchain-based asset management approach are assessed to determine its efficacy.

The second stage focuses on asset management within the nuclear energy infrastructure. This stage begins with evaluating the need for more efficient asset management practices. The evaluation considers the current state of asset management, identifying areas where blockchain technology could enhance operations. If the need is established, a blockchain-based asset management system is implemented. This system is designed to record comprehensive data on asset ownership, maintenance schedules, and compliance with regulatory requirements. By leveraging blockchain technology, the system aims to improve efficiency and transparency in managing nuclear assets. The data management capabilities of blockchain ensure that all information is accurate, immutable, and easily accessible. The effectiveness of the blockchain-based asset management system is then evaluated based on cost-effectiveness, operational efficiency, and transparency improvements. The procedure advances to Energy Trading & Grid Management, the following step, if the system is found to be efficient.

### 4.3 Energy trading & grid management

Energy trade and grid management become the main topics of discussion in the third stage. Assessing if peer-to-peer energy trading is required in the nuclear energy industry is the first stage. The assessment entails scrutinizing the possible advantages of this type of trading system, comprising heightened market involvement and enhanced grid functionalities. A system based on blockchain technology is put in place to enable peer-to-peer energy trade if it is determined to be advantageous. The system's goal is to maximize grid performance and guarantee fair pricing by facilitating secure, transparent transactions across energy providers and consumers. Transparency and accountability are provided by the blockchain technology, which guarantees that every transaction is documented in an encrypted and unchangeable ledger. The market participation, cost-effectiveness, and operational efficiency of the blockchain-based energy trading system are then used to evaluate its efficiency. If the system appears to be functioning well, the next step in the process is regulatory compliance.

### 4.4 Regulatory compliance

In the nuclear energy sector, regulatory compliance is the focus of the fourth stage. The first step in this approach is to assess if reporting and verification procedures need to be shortened. The assessment looks at the legal system as it is and pinpoints sectors where the application of blockchain technology could improve compliance. A blockchain-based solution is put into place if it is determined that better regulatory procedures are required. This system's goal is to simplify reporting and verification procedures so that businesses may more easily adhere to legal obligations. Blockchain technology improves regulatory supervision and auditability by ensuring that all information related to regulation is recorded in a transparent and safe manner. Subsequently, the efficacy of the blockchain-driven regulatory compliance framework is assessed by considering the decrease in regulatory burden, heightened transparency, and enhanced auditability. The procedure advances to the next phase, Nuclear Safeguards, if the system is found to be successful.

### 4.5 Nuclear safeguards

The emphasis of the following stage is nuclear safeguards, with the first step being to ascertain if auditable records of actions within the nuclear industry are required. The benefits of keeping thorough and secure records are examined, along with the possible concerns of diversion and proliferation. A system that utilizes the blockchain is put into place if it is determined that auditable documents are necessary. In order to lower the possibility of proliferation and diversion, this system is made to keep complete and unchangeable documents of all nuclear activities. All records are safe, open, and simple to audit thanks to blockchain technology. Next, the security, transparency, and accountability aspects of the blockchain-based nuclear safeguards system are assessed. The following step of the process, Decentralized Energy Systems, is where the system goes if it seems to be successful.

### 4.6 Decentralized energy systems

In the sixth stage, nuclear energy is integrated with decentralized energy systems, which also include storage and renewable energy sources. Taking into account the possible advantages of improved energy resilience and sustainability, the first stage is to evaluate the necessity of such integration. A blockchain-based system is put into place if it is determined that integration is necessary. In order to promote energy resilience and sustainability, this technology is made to make it easier to integrate nuclear energy with storage options and renewable energy sources. Coordination and efficiency are improved since blockchain technology makes sure that every integration step is transparently and securely documented. Then, based on integration productivity, cost savings, and sustainability benefits, the efficacy of the blockchain-based decentralized energy systems is assessed. In the event that the system works as intended, the procedure moves on to problems and their fixes.

### 4.7 Security challenges and solutions

Continuous consideration and resolution of persistent issues including data protection, system interoperability, and regulatory compliance are crucial throughout the whole process. For blockchain technology to be successfully integrated into the nuclear energy industry, these issues must be carefully considered, and workable solutions must be developed. New legislative frameworks, improved data privacy safeguards, and interoperability between blockchain systems are a few potential solutions. In order to significantly increase efficiency, transparency, security, and sustainability in the nuclear energy industry, the overarching purpose of this strategy implementation is to fully utilize blockchain technology. The industry can create a more reliable, safe, and future-proof energy infrastructure by methodically addressing each step and resolving related obstacles.

### 4.8 Limitations

While the significant interconnection between blockchain and IoT technologies has been explored in our study. We have utilized through a range of applications, privacy and security issues, possible fixes, and pertinent algorithms. We have also looked at how Blockchain technology may be used in the nuclear industry. We specifically looked at "Cryptographic Secure Transaction Process in Blockchain," "IoT Applications and Data Flow Framework," "Secure Data Management Framework," "Security and Privacy Challenges in Blockchain-IoT Integration," and "Unveiling the Power of Blockchain and IoT." It is crucial to recognize several limitations that are intrinsic to the current investigation.

• **Theoretical framework:** The main emphasis of our research is on a theoretical framework for blockchain-IoT integration-based safe data management in nuclear energy. Although this framework offers a useful starting point, more verification via pilot applications or simulations in regulated nuclear energy scenarios is required to evaluate its practicality.
• **Considerations for implementation:** Using blockchain technology to implement a secure data management framework in IoT devices with limited resources may cause processing lags or energy consumption issues. To verify that the framework is feasible in resource-constrained environments, further research might investigate optimization techniques to reduce these possible downsides.
• **Security analysis scope:** Certain security and privacy issues pertaining to Blockchain-IoT integration may be given priority in the research. It's crucial to recognize that new and developing cyberthreats may necessitate regular vulnerability assessments. Because cyber threats are always evolving, security mechanisms inside the framework must also be continuously improved.
• Data availability: The availability of real-time data on privacy and security violations in nuclear energy deployments may be restricted by security measures. This could make it more difficult to thoroughly assess how successful the suggested fixes would be in a practical setting. Additional investigation into controlled conditions or the use of synthetic or anonymized data may yield insightful information that helps to improve the framework.

The preceding constraints underscore the necessity for more investigation to close the knowledge gap between conceptual models and practical applications in the nuclear industry.

## 5 Conclusion

This study investigated the potential of integrating blockchain and IoT technologies to enhance the privacy and security of data management framework within the nuclear energy sector. Our finding highlighted the significant benefits of this integration: blockchain's immutability and transparency property offer robust data integrity and validation, while IoT's real-time data collecting capabilities provides data monitoring and evaluation of vital systems. However, the study also highlighted the challenges associated with scalability, security, privacy and integrity concerns due to the decentralized nature of the blockchain. To address these challenges, we have illustrated the integration framework and proposed the salutation to mitigate security and privacy concerns. We also introduced an IoT application architecture tailored for secure blockchain-based data management in the nuclear energy sector. Overall, this study shows how blockchain and IoT integration may be used to secure data in the nuclear energy industry. Researchers and practitioners may work toward achieving this integration in a secure and effective manner by addressing the difficulties that have been highlighted and utilizing the framework and solutions that have been suggested. By demonstrating the feasibility of this approach within the nuclear energy context, our research contributes to the advancement of secure and reliable critical infrastructure systems.

## 6 Future scope

Expanding upon our evaluation of integration of blockchain and IoT technologies, future studies focus on many crucial domains that will address the limitations highlighted in our study. To evaluate the theoretical framework's viability, it must first be validated in practical circumstances using pilot implementations or simulations of controlled nuclear energy scenarios. Furthermore, research should concentrate on ways to reduce latency and energy consumption problems in order to optimize blockchain implementation for IoT devices with limited resources. Regular vulnerability evaluations and ongoing security mechanism development are essential for maintaining adequate security considering the dynamic nature of cyberthreats. In addition, resolving issues with data availability through the use of synthetic and anonymized data or controlled conditions can aid in a more complete assessment of the efficacy of proposed methodology. These steps have significance for bridging the gap between theoretical models and practical implementations, therefore enhancing the practical integration of blockchain and IoT in the nuclear sector.

## Funding

This research received no external funding.

## Data availability statement

The data used in this study are reported in the paper's figures and tables.

## CRediT authorship contribution statement

**Hari Mohan Rai:** Writing – original draft, Visualization, Validation, Supervision, Resources, Investigation, Conceptualization. **Kaustubh Kumar Shukla:** Writing – original draft, Investigation, Conceptualization. **Lilia Tightiz:** Writing – original draft, Investigation. **Sanjeevikumar Padmanaban:** Writing – original draft, Supervision, Investigation, Funding acquisition, Conceptualization.

## Declaration of competing interest

The authors declare that they have no known competing financial interests or personal relationships that could have appeared to influence the work reported in this paper.
